The article "Study on the Effect of Positive Psychological Intervention Based on PERMA Model on Perioperative Patients with AIDS Complicated with Breast Cancer" was published in 2022. Journal: Comput Math Methods Med.

# Study on the Effect of Positive Psychological Intervention Based on PERMA Model on Perioperative Patients with AIDS Complicated with Breast Cancer

**DOI:** 10.1155/2022/9788122

**Published:** 2022-08-08

**Authors:** Lingmei Luo, Ying Li, Zhou Zhou, Saifen Yang, Yao Qin, Hua Peng, Yirong Wang, Zhe Li, Tianqin Yin

**Affiliations:** Department of Infectious Diseases Surgery, The First Hospital of Changsha, Changsha, Hunan Province 410000, China

## Abstract

**Objective:**

To study the effect of positive psychological intervention based on PERMA model on perioperative AIDS patients complicated with breast cancer.

**Methods:**

A total of 120 perioperative patients with AIDS complicated with breast cancer treated in our hospital from January 2021 to December 2021 were randomly divided into research group (*n* = 60) and control group (*n* = 60). The research group received positive psychological intervention based on PERMA model, while the control group received routine nursing. The scores of disease uncertainty scale (MUIS), Frankl treatment compliance scale, cancer-related fatigue scale, self-rating anxiety scale (SAS), self-rating depression scale (SDS), and quality of life scale EORTCQLQ-C30 (v3.0) were studied.

**Results:**

After 12-week nursing, the MUIS score of the research group was lower than that of the control group, and the difference was statistically significant (*P* < 0.05). After 12 weeks of nursing, the score of Frankl treatment compliance scale in the research group was higher than that in the control group, and the difference was statistically significant (*P* < 0.05). Following 12-week nursing, the scores of SAS and SDS in the research group were lower than those in the control group, and the difference was statistically significant (*P* < 0.05). After 12 weeks of nursing, the score of cancer-related fatigue scale in the research group was lower than that in the control group, and the difference was statistically significant (*P* < 0.05). The EORTCQLQ-C30 (v3.0) scale-symptom domain score in the research group was lower than that in the control group following 12-week nursing, and the difference was statistically significant (*P* < 0.05). After 12 weeks of nursing, the EORTCQLQ-C30 (v3.0) scale-overall health domain score and functional domain score in the research group were higher than those in the control group, and the difference was statistically significant (*P* < 0.05).

**Conclusion:**

The application value of positive psychological intervention based on PERMA model in perioperative patients with AIDS complicated with breast cancer is more significant. It contributes more to treatment compliance and improves negative feelings of anxiety and depression.

The article "Study on the Effect of Positive Psychological Intervention Based on PERMA Model on Perioperative Patients with AIDS Complicated with Breast Cancer" was published in 2022. Journal: Comput Math Methods Med.

## 1. Introduction

Acquired immunodeficiency syndrome (AIDS) is a highly contagious infectious disease caused by human immunodeficiency caused by human infection with human immunodeficiency virus (HIV) [1]. AIDS cannot be cured, because HIV specifically invades human CD4^+^ cells, causing serious damage to the human immune system. By the end of 2017, there were 36.9 million people living with HIV worldwide, of which 1.8 million were new HIV infections [2]. In China, as a country with a large population, the number of new AIDS patients is also very staggering. From 2012 to 2017, the number of new cases of HIV/AIDS in China increased from 82434 to 134512 every year and there is still an upward trend [3, 4]. According to the latest data of the Chinese Center for Disease Control and Prevention, there were 445716 cases of HIV infection and 323456 cases of AIDS in China by the end of January 2018 with 241519 reported deaths [5]. The widespread spread of AIDS has become a serious social problem.

AIDS patients with depression need effective psychological intervention and support to ensure the effectiveness and health of nursing measures. A large number of foreign studies have examined the effect of psychological intervention on AIDS patients from an empirical point of view, which is effective in immune function, emotional regulation, compliance, and high-risk sexual transmission blocking. According to clinical studies, a large number of AIDS patients suffer from malignant tumors. Before 1995, AIDS-related malignant tumors such as Kaposi's sarcoma, non-Hodgkin's lymphoma, and invasive cervical cancer accounted for 80% of the total cancer burden of AIDS patients [6, 7]. In recent years, due to the improvement of the level of antiretroviral therapy and the level of minimally invasive breast surgery, the survival rate of AIDS patients with breast cancer has also been effectively improved [8]. However, AIDS patients with breast cancer still need to face various problems such as social discrimination, economic, and mental pressure. AIDS combined with breast cancer not only seriously damages the life and health of patients but also brings more serious psychological trauma to patients [9, 10]. Numerous studies have pointed out that psychological intervention can play an important and positive role in the maintenance of AIDS and mental health [11–13]. With the popularization of treatment, the proportion of malignant tumors in AIDS patients has changed greatly and the proportion of non-HIV-related malignant tumors such as breast cancer has increased significantly [14–17]. PERMA model is a happiness model proposed by Seligman, which consists of five elements such as positive emotion, input, interpersonal relationship, meaning, and achievement. The theory holds that having these five elements can overcome negative emotions and have a happy life [18]. At present, PERMA model has been used in stroke disabled patients [19], AIDS hospitalized patients [20], disabled college students [21], and achieved good results, but it is not known whether this model is suitable for perioperative AIDS patients with breast cancer in China. Therefore, this paper studied the effect of positive psychological intervention based on PERMA model on perioperative patients with AIDS complicated with breast cancer.

The article "Study on the Effect of Positive Psychological Intervention Based on PERMA Model on Perioperative Patients with AIDS Complicated with Breast Cancer" was published in 2022. Journal: Comput Math Methods Med.

## 2. Materials and Methods

### 2.1. General Information

A total of 120 perioperative AIDS patients with breast cancer treated in our hospital from January 2021 to December 2021 were selected. 120 perioperative AIDS patients with breast cancer were randomly divided into research group (*n* = 60) and control group (*n* = 60). In the research group, the age ranged from 25 to 67 years old with an average of 54.48 ± 5.16 year old. In the control group, the age ranged from 25 to 68 years old with an average of 54.15 ± 5.33 years old. There was no significant difference in general data between the two groups (*P* > 0.05).

Inclusion criteria are as follows: (1) female patients with primary breast cancer who met the indications for surgical treatment; (2) hospitalized patients diagnosed with AIDS; (3) those who had access to the Internet and were proficient in using WeChat; (4) their condition was basically stable and can basically take care of themselves. No special hobbies such as drug use and alcohol abuse; (5) normal spirit and intelligence and normal communication skills such as listening, speaking, reading, and writing; and (6) volunteer to participate in this study.

Exclusion criteria are as follows: (1) with other cancers or serious basic diseases such as heart, liver, and kidney; (2) mental illness or disturbance of consciousness; (3) cases with low intelligence did not have basic listening, speaking, reading, and writing skills; (4) patients who were unable to care for themselves; (5) cases with mental illness, paranoid personality, drug addicts, and alcoholics; and (6) cases without Internet access and will not use WeChat, QQ, and other chat tools.

### 2.2. Methods

#### 2.2.1. Technical Route

Figure 1 shows the technology roadmap.

#### 2.2.2. Intervention Scheme

Control group scheme: routine care: from the first week of hospitalization, the responsible nurse conducted 8 consecutive health education interviews with the patients, including the following: (1) introduction and prevention of AIDS and breast cancer, (2) introduction and countermeasures of common complications of AIDS, (3) introduction of common programs for antiviral treatment of AIDS, (4) introduction of breast cancer operation plan, (5) medication guidance and common adverse drug reactions of AIDS complicated with breast cancer, (6) dietary guidance, (7) compliance education of antiviral drugs, (8) the significance and indication of perioperative prophylactic medication, and (9) the present situation and prospect of antiretroviral therapy and minimally invasive breast surgery. The WeChat group was established to keep in touch with patients and to encourage patients to continue to participate in the study. If the patient was discharged, the patient would be interviewed through WeChat voice chat, message, or phone.

The article "Study on the Effect of Positive Psychological Intervention Based on PERMA Model on Perioperative Patients with AIDS Complicated with Breast Cancer" was published in 2022. Journal: Comput Math Methods Med.

Research group plan: the research group was given positive psychological intervention based on PERMA model. One phase was 3 weeks, 4 phases, a total of 12 weeks. The first three stages were intervened twice, and the last stage intervention only needed once with a total of 7 times. Every time 30~50 min, the intervention place was the breast surgery demonstration room. The intervention methods were interviews and exercises, including on-site guidance and home-based exercises. The specific contents included (1) the first time: Interviews were conducted with patients around their feelings after the illness. The patient was asked to talk about his negative thoughts and to guide the patient to think dialectically about the idea. (2) The second time is as follows: to introduce positive emotion. The patients were guided to understand and familiarize themselves with the relevant knowledge of positive emotions and to conduct preliminary exercises on positive emotions. Through the combination of slides and videos, the famous experiments of positive psychology were introduced to patients in an easy-to-understand language. The interviews with patients would be conducted around people or things that needed to be grateful during illness. (3) The third time is as follows: to establish positive emotion. The patients were guided to cultivate positive thinking and interviewed around positive events in life. (4) The fourth time is as follows: to input. The patients were guided to understand and familiarize themselves with the relevant knowledge of input and flow experience. The patients were encouraged to conduct preliminary exercises on flow experience interview content. (5) The fifth time is as follows: relationship. The patients were guided to understand and be familiar with the relevant knowledge of interpersonal communication methods and skills. (6) The sixth time is as follows: meaning. Guided patients were asked to understand and familiarize themselves with the relevant knowledge of the meaning of life. The patients should find and determine their own meaning of life interview content through the combination of slides and videos to introduce real examples of meaningful life to patients. (7) The 7th time is as follows: goals and achievements. The patients were informed and familiarized with goals and achievements. The patients were guided to set goals that are of interest to them. The patients were presented with real-life examples of discharged patients' achievements through a combination of slides and videos.

The article "Study on the Effect of Positive Psychological Intervention Based on PERMA Model on Perioperative Patients with AIDS Complicated with Breast Cancer" was published in 2022. Journal: Comput Math Methods Med.

### 2.3. Observation Index

1. *Mishel Uncertainty in Illness Scale (MUIS)*. The total score of MUIS ranged from 320 to 160.
2. *Frankl Treatment Compliance Scale*. The scoring criteria of Frankl compliance scale were as follows: 1: refusal, pain; 2: uncooperation, reluctance; 3: use, indifference; and 4: active cooperation and enjoyment.
3. The scores of self-rating anxiety scale (SAS) and self-rating depression scale (SDS) were studied. Anxiety was defined as the standard score of SAS ≥ 50. With the increase of the score, the degree of anxiety was more serious. The standard score of SDS ≥ 53 points was seen as depression.
4. *The Score of Cancer-Related Fatigue Scale*. The scale of cancer-related fatigue includes behavioral fatigue, cognitive fatigue, physical fatigue, and emotional fatigue with a full score of 10.
5. The EORTCQLQ-C30 (v3.0) score of the quality-of-life measurement scale was studied. The EORTCQLQ-C30 (v3.0) scale included a total of 15 evaluation dimensions and 30 items. The functional areas were included: 5 items of body, 2 items of role, 2 items of cognition, 4 items of emotion, and 2 items of social function; general health status is as follows: 1 item of general health and 1 item of quality of life. The domain (12 items for fatigue, pain, nausea, and vomiting and 1 item for health-related economic conditions) had a total of 30 items. Among them, items 29 and 30 were scored on the scale of 1-7 points, while the others were scored on the order of 1-4 points.

### 2.4. Statistical Analysis

The IBMSPSS24.0 software was applied for statistical analysis. The measurement data were expressed by mean ± standard deviation. The counting data were expressed by frequency or rate. *t*-test was used when measurement data obey normal distribution, and rank sum test was used when it did not obey normal distribution. *χ*^2^ test was used to compare the classified counting data. Repeated measurement data were analyzed by repeated measurement analysis of variance. Main effect test results were used when there was no interaction, and simple effect analysis was carried out when there was interaction. *P* < 0.05 indicated that the difference between groups is statistically significant.

The article "Study on the Effect of Positive Psychological Intervention Based on PERMA Model on Perioperative Patients with AIDS Complicated with Breast Cancer" was published in 2022. Journal: Comput Math Methods Med.

## 3. Results

### 3.1. The Score of MUIS

Before nursing, there was no significant difference in the MUIS score between the two groups (*P* > 0.05). After 12 weeks of nursing, the MUIS score in the research group was lower than that in the control group, and the difference was statistically significant (*P* < 0.05) (see Table 1).

### 3.2. Study Frankl Scale Score

Before nursing, there was no significant difference in the scores of Frankl scale between the two groups (*P* > 0.05). After 12 weeks of nursing, the scores of Frankl scale in the research group were higher than those in the control group, and the difference was statistically significant (*P* < 0.05) (see Table 2).

### 3.3. The Score of SAS and SDS

Before nursing, the SAS and SDS scores of the two groups were not statistically significant (*P* > 0.05). After 12 weeks of nursing, the SAS and SDS scores of the research group were lower than those of the control group, and the difference was statistically significant (*P* < 0.05) (see Table 3).

### 3.4. The Score of Cancer-Related Fatigue Scale

Before nursing, there was no significant difference in the score of cancer-related fatigue scale between the two groups (*P* > 0.05). However, the score of cancer-related fatigue scale in the research group was lower than that in the control group following 12-week nursing, and the difference was statistically significant (*P* < 0.05) (see Table 4).

### 3.5. Study the Score of EORTC QLQ-C30 (v3.0) Scale

Before nursing, there was no statistical difference in the scores of EORTCQLQ-C30 (v3.0) between the groups (*P* > 0.05). After 12 weeks of nursing, the EORTCQLQ-C30 (v3.0) scale-symptom domain score of the research group exhibited lower than the control group, and the difference was statistically significant (*P* < 0.05). After 12 weeks of nursing, the EORTCQLQ-C30 (v3.0) scale-general health domain score and functional domain score of the research group were higher than those of the control group, and the difference was statistically significant (*P* < 0.05) (see Table 5).

## 4. Discussion

Clinical studies have shown that HIV mainly invades host CD4+ cells (T cells, mononuclear macrophages, dendritic cells, etc.). It can bind to the CD4 molecule on the surface of the target cell membrane through the glycoprotein glp20 of its outer membrane. In addition, glp20-CD4 is able to bind to the chemokine receptor CXCR4 or CCR5 expressed on the surface of the target cell membrane to form a trimolecular complex of CD4-glp20-CCR5 (or CCR4), which will result in the conformational change of glp20 and exposes the masked gp41. gp41 is capable of inserting directly into the target cell membrane. The hydrophobic effect of the membrane itself mediated the fusion of the virus envelope and the cell membrane, which makes the virus enter the target cells and directly damage the immune defense and immune surveillance function [22]. CXCR4 receptor not only exists on the surface of CD4+ T cells but also highly expressed on the surface of breast cancer cells. A large number of studies have proved that the combination of breast cancer cell CXCR4 and its ligand CXCL12 can promote the proliferation of primary tumor and distant metastasis of liver, lung, and brain, which will aggravate the patient's condition and increase the difficulty of treatment [23]. Therefore, there is a certain association between AIDS breast cancer. Many patients are suffering from these two diseases at the same time.

The article "Study on the Effect of Positive Psychological Intervention Based on PERMA Model on Perioperative Patients with AIDS Complicated with Breast Cancer" was published in 2022. Journal: Comput Math Methods Med.

The treatment of breast cancer has the characteristics of diversity and combination, and local treatment includes surgical resection, local radiotherapy, systemic therapy including chemotherapy, endocrine therapy, and targeted therapy [24]. AIDS patients with breast cancer are more likely to have serious mental and psychological problems such as anxiety and depression. Applying positive psychological intervention based on PERMA model to breast cancer patients can reduce the fear of cancer recurrence in breast cancer patients [25].

Due to the chronic incurability of AIDS and public panic and discrimination against AIDS, people with AIDS are more likely to suffer from many psychological problems, such as anxiety, depression, discrimination, guilt, and suicidal tendencies [26]. Shurong conducted a questionnaire survey on 321 newly diagnosed HIV infections and found that the positive rates of depressive symptoms, anxiety symptoms, and suicidal ideation were 41.1% (132/321), 31.5% (101/321), and 27.7% (89/321), respectively [27]. Early findings have shown that AIDS patients with depression need additional psychological intervention and support from health care interventions [28]. However, the nurses in our country have a low mastery of psychological nursing knowledge, and the application of psychological nursing in AIDS patients is very rare [29]. The only psychological nursing research is only in the exploratory stage [30–34]. Thus, the current psychological care cannot meet the psychological needs of AIDS patients. Some studies have shown that the application of positive psychological intervention based on PERMA model to AIDS patients can improve the subjective well-being of AIDS patients [35]. Among AIDS patients, there is no lack of patients with low BMI and poor nutritional status. The immune function is impaired, and the adverse reactions caused by chemotherapeutic drugs are more obvious. As a result, the cancer progression of AIDS patients is faster than that of the general population, so the prognosis of AIDS patients with breast cancer is poor, which not only requires our active treatment [36, 37]. Therefore, this study introduced positive psychological intervention based on PERMA model into perioperative nursing care of AIDS patients with breast cancer.

The article "Study on the Effect of Positive Psychological Intervention Based on PERMA Model on Perioperative Patients with AIDS Complicated with Breast Cancer" was published in 2022. Journal: Comput Math Methods Med.

The results of this study proved that the application value of positive psychological intervention based on PERMA model in perioperative patients with AIDS complicated with breast cancer is more significant. It is more helpful to reduce the uncertainty of disease and the degree of cancer-related fatigue. This is mainly because the incidence of anxiety and depression in AIDS is high [37]. Some studies have shown that the ability of emotion adjustment plays a very important role in controlling the occurrence and development of anxiety and depression in AIDS patients. It is also an important index to evaluate mental health [38]. In the PERMA model, clinical medical staff should include positive psychological factors such as emotion, input, interpersonal relationship, meaning, and achievement in the health guidance management system of AIDS patients with breast cancer [39, 40]. In the guidance of propaganda and education, more attention should be paid to the psychological status of patients. Furthermore, their negative emotions such as anxiety and depression should be reduced through the training of positive explanation and optimistic explanation style in the interview. It can increase the positive emotion through gratitude practice, the establishment of positive emotion file, and the improvement of interpersonal relationship by active response, so as to guide patients to express their negative emotion towards the disease. Specific negative psychological aspects of the patient are identified, and counselling and thought-transformation exercises are given to help patients change their negative perceptions of the illness, reduce their uncertainty about the illness, and enhance their positive emotions and experiences. In addition, the patients are made to understand that their current negative emotions are related to misperceptions through the principles of cognitive intervention. Through the further understanding of the disease, the patients will learn to explain the current physical problems and challenges from a positive point of view, which greatly increases their confidence in resisting the disease. There are some limitations in this study. First, the sample size of this study is not large, and it is a single-center study, so bias is inevitable. In future research, we will carry out multicenter, large-sample prospective studies, or more valuable conclusions can be drawn.

The article "Study on the Effect of Positive Psychological Intervention Based on PERMA Model on Perioperative Patients with AIDS Complicated with Breast Cancer" was published in 2022. Journal: Comput Math Methods Med.

In conclusion, the application value of positive psychological intervention based on PERMA model in perioperative patients with AIDS complicated with breast cancer is more significant. It is more helpful to reduce disease uncertainty and cancer-related fatigue and, in the meanwhile, to improve treatment compliance and quality of life.

## Figures and Tables

**Figure 1:** Technology roadmap.

**Table 1:** MUIS score ($\bar{x}\pm s$, points).

Grouping	*N*	Before nursing (points)	After 12 weeks of nursing (points)
Control group	60	59.53 ± 6.14	41.15 ± 3.27^∗^
Research group	60	59.45 ± 6.23	36.19 ± 2.04^∗^
*t* value		0.071	9.968
*P* value		0.945	<0.01

Note: ∗ represented the comparison of this group before nursing and 12 weeks after nursing, and the difference was statistically significant (*P* < 0.05).

**Table 2:** Frankl treatment adherence scale scores ($\bar{x}\pm s$, points).

Grouping	*N*	Before nursing	After 12 weeks of nursing
Control group	60	1.24 ± 0.31	2.69 ± 0.28^∗^
Research group	60	1.21 ± 0.32	3.69 ± 0.08^∗^
*t* value		0.522	26.599
*P* value		0.603	<0.01

Note: ∗ represented the comparison of this group before nursing and 12 weeks after nursing, and the difference was statistically significant (*P* < 0.05).

**Table 3:** The score of SAS and SDS ($\bar{x}\pm s$, points).

Grouping	N	SAS scoring		SDS scoring	
		Before nursing	After 12 weeks of nursing	Before nursing	After 12 weeks of nursing
Control group	60	66.34 ± 5.32	57.66 ± 4.08^∗^	72.45 ± 7.26	62.23 ± 6.14^∗^
Research group	60	66.29 ± 5.45	50.44 ± 3.25^∗^	72.38 ± 7.34	50.29 ± 2.03^∗^
*t* value		0.051	10.722	0.053	14.302
*P* value		0.959	<0.01	0.958	<0.01

Note: ∗ represented the comparison of this group before nursing and 12 weeks after nursing, and the difference was statistically significant (*P* < 0.05).

**Table 4:** The score of cancer-related fatigue scale ($\bar{x}\pm s$, points).

Grouping	*N*	Before nursing	After 12 weeks of nursing
Control group	60	8.59 ± 1.17	6.36 ± 0.25^∗^
Research group	60	8.63 ± 1.14	4.02 ± 0.12^∗^
*t* value		0.189	65.362
*P* value		0.849	<0.01

Note: ∗ represented the comparison of this group before nursing and 12 weeks after nursing, and the difference was statistically significant (*P* < 0.05).

**Table 5:** EORTC QLQ-C30 (v3.0) scale score ($\bar{x}\pm s$, points).

Grouping	*N*	Symptom field		Functional area	General health field		
		Before nursing	After 12 weeks of nursing	Before nursing	After 12 weeks of nursing	Before nursing	After 12 weeks of nursing
Control group	60	36.44 ± 3.28	29.59 ± 2.32^∗^	15.54 ± 2.09	25.39 ± 4.13^∗^	3.15 ± 0.25	4.03 ± 0.45^∗^
Research group	60	36.12 ± 3.34	24.36 ± 1.14^∗^	15.65 ± 2.02	40.77 ± 5.12^∗^	3.16 ± 0.08	7.12 ± 0.11^∗^
*t* value		0.529	15.672	0.293	18.111	0.295	51.668
*P* value		0.598	<0.01	0.769	<0.01	0.768	<0.01

Note: ∗ represented the comparison of this group before nursing and 12 weeks after nursing, and the difference was statistically significant (*P* < 0.05).

The article "Study on the Effect of Positive Psychological Intervention Based on PERMA Model on Perioperative Patients with AIDS Complicated with Breast Cancer" was published in 2022. Journal: Comput Math Methods Med.

## Data Availability

No data were used to support this study.

## References

[1] Koski L., Brouillette M. J., Mayo N. E., Scott S. C., Fellows L. K., Sookman D. (2022). A short-term psychological intervention for people living with HIV during the first wave of COVID-19. *International Journal of Cognitive Therapy*.

[2] Ajayi A. I., Mudefi E., Adeniyi O. V., Goon D. T. (2019). Achieving the first of the joint United Nations Programme on HIV/AIDS (UNAIDS) 90-90-90 targets: understanding the influence of HIV risk perceptions, knowing one’s partner’s status and discussion of HIV/sexually transmitted infections with a sexual partner on uptake of HIV testing. *International Health*.

[3] Ruijuan L. (2020). The value of high quality nursing when nursing breast cancer patients with arm TIVAP. *Chinese community physician*.

[4] STD Control Center of Chinese Center for Disease Control and Prevention (2018). National AIDS/STD epidemic situation in December 2017. *AIDS and sexually transmitted diseases in China*.

[5] STD Control Center of China Center for Disease Control and Prevention (2018). January 2018 national AIDS and STD epidemic situation. *AIDS and sexually transmitted diseases in China*.

[6] Foschiera L. N., Dupont M. F., Habigzang L. F. (2022). Follow-up evaluation of psychotherapy protocols for women with a history of intimate partner violence: scoping review. *Trends in Psychology*.

[7] Hong X. (2018). Self-confidence group psychological intervention of college students based on EEG test technology-take patients with social anxiety disorder as an example. *Neuro Quantology*.

[8] Rebeiro P. F., Mcpherson T. D., Goggins K. M. (2018). Health literacy and demographic disparities in HIV care continuum outcomes. *AIDS and Behavior*.

[9] Pramod S. (2021). A soft silicone foam dressing that aids healing and comfort in oncology care. *British journal of nursing (Mark Allen Publishing)*.

[10] Fei J., Xiuling F., Ruiyin Z. (2021). Effects of preservation of anterior thoracic nerve and intercostobrachial nerve on postoperative recovery and incidence of complications in patients undergoing radical mastectomy. *Clinical Medicine*.

The article "Study on the Effect of Positive Psychological Intervention Based on PERMA Model on Perioperative Patients with AIDS Complicated with Breast Cancer" was published in 2022. Journal: Comput Math Methods Med.

[11] Glick J. L., Russo R., Jivapong B. (2020). The PrEP care continuum among cisgender women who sell sex and/or use drugs globally: a systematic review. *AIDS and Behavior*.

[12] Emery J. D., Nguyen P., Minshall J., Cummings K. L., Walker J. (2018). Chemoprevention: a new concept for cancer prevention in primary care. *Australian journal of general practice*.

[13] Haberl L., Audebert F., Feiterna-Sperling C. (2021). Not recommended, but done: breastfeeding with HIV in Germany. *AIDS Patient Care and STDs*.

[14] Kristin B. S., Begnel E. R., Golden M. R., Moore A., Ramchandani M., Dombrowski J. C. (2020). "It's me as a person, not me the disease": patient perceptions of an HIV care model designed to engage persons with complex needs. *AIDS Patient Care and STDs*.

[15] Haque R., Chlebowski R. T., Chen L. H. (2021). Sleep medication use and risk of fractures in breast cancer survivors. *Breast Cancer Research and Treatment*.

[16] Camacho F., Anderson R., Kimmick G. (2019). Investigating confounders of the association between survival and adjuvant radiation therapy after breast conserving surgery in a sample of elderly breast cancer patients in Appalachia. *BMC Cancer*.

[17] Zdenkowski N., Butow P., Spillane A. (2018). Single-arm longitudinal study to evaluate a decision aid for women offered neoadjuvant systemic therapy for operable breast cancer. *Journal of the National Comprehensive Cancer Network: JNCCN*.

[18] Howell L. P., DeNardo S. J., Levy N. B., Lund J., Denardo G. L. (2018). Immunohistochemical staining of metastatic ductal carcinomas of the breast by monoclonal antibodies used in imaging and therapy: a comparative study. *The International Journal of Biological Markers*.

[19] Gao J. P., Jin Y. H., Yu S. F., Wu W. F., Han S. F. (2021). Evaluate the effectiveness of breast cancer decision aids: a systematic review and meta-analysis of randomize clinical trails. *Nursing Open*.

[20] Si J., Guo R., Lu X. (2020). Decision aids on breast conserving surgery for early stage breast cancer patients: a systematic review. *BMC Medical Informatics and Decision Making*.

[21] Yu L., Li P., Yang S. (2020). Web-based decision aids to support breast cancer screening decisions: systematic review and meta-analysis. *Journal of Comparative Effectiveness Research*.

[22] Yao K., Belkora J., Lee C. (2019). An in-visit decision aid for surgeons to address decision making for bilateral mastectomy for newly diagnosed breast cancer patients. *Annals of Surgical Oncology*.

[23] Gocko X., Fondacci M., Dibi C., Plotton C. (2020). Information around organized breast cancer screening. Do INCa and Cancer Rose meet criteria for decision aids?. *Revue d'epidemiologie et de sante publique*.

The article "Study on the Effect of Positive Psychological Intervention Based on PERMA Model on Perioperative Patients with AIDS Complicated with Breast Cancer" was published in 2022. Journal: Comput Math Methods Med.

[24] Anbari A. B., Ostby P., Ginex P. K. (2020). Breast cancer–related lymphedema: personalized plans of care to guide survivorship. *Current Breast Cancer Reports*.

[25] Kimmel A. D., Masiano S. P., Bono R. S. (2018). Structural barriers to comprehensive, coordinated HIV care: geographic accessibility in the US south. *AIDS Care*.

[26] Yudan L. (2018). Study on the application of cognitive behavioral therapy combined with sleep intervention nursing in postoperative chemotherapy of breast cancer patients. *World Journal of Sleep Medicine*.

[27] Shurong Y. (2021). To explore the clinical application of surgical rapid rehabilitation concept in nursing perioperative patients with breast cancer after modified radical mastectomy. *Intelligence and health*.

[28] Hal G. V., Garcia P. D. (2021). Lung cancer screening: targeting the hard to reach—a review. *Translational Lung Cancer Research*.

[29] Lin S. (2020). To explore the effect of rapid rehabilitation surgery in nursing perioperative patients with breast cancer after modified radical mastectomy. *Chinese Medicine Guide*.

[30] Lijun H. (2019). Observation on the perioperative clinical effect of psychological nursing for patients with breast cancer. *Chinese Medicine Guide*.

[31] Mccrorie A. D., Begley A. M., Chen J. J., McCorry N. K., Paget G., McIntosh S. A. (2021). Improving preparedness prior to reconstructive breast surgery via inclusion of 3D images during pre-operative counselling: a qualitative analysis. *BMC Women's Health*.

[32] Zhili Z. (2018). Application of rapid rehabilitation surgery concept in nursing perioperative patients with breast cancer after modified radical mastectomy. *Everyone's Health (mid-edition)*.

[33] Jianping W. (2018). Improvement of blood hypercoagulable state of patients with breast cancer after radical mastectomy by comprehensive rehabilitation nursing of traditional Chinese medicine. *Thrombus and hemostasis*.

[34] Lixiang C. (2018). Observation on the effect of standardized skin care on skin lesions of breast cancer after radiotherapy. *Bethune Medical Journal*.

[35] Kern M. L., Waters L. E., Adler A., White M. A. (2015). A multidimensional approach to measuring well-being in students: Application of the PERMA framework. *The journal of positive psychology*.

[36] Vishnuteja M., Rout S. S., Sahoo P. K. (2021). A prospective study of triple assessment in evaluation of breast lump. *International Journal of Advanced Research*.

[37] Chunhao X. (2018). Effect of intervention nursing on cancer-related fatigue and quality of life in breast cancer patients undergoing chemotherapy. *Chinese and foreign medical research*.

[38] Weina X., Lin P. (2018). Explore the effect of routine nursing and aerobic exercise combined with music therapy in postoperative nursing of breast cancer. *Contemporary medicine*.

The article "Study on the Effect of Positive Psychological Intervention Based on PERMA Model on Perioperative Patients with AIDS Complicated with Breast Cancer" was published in 2022. Journal: Comput Math Methods Med.

[39] Sadeghi M., Farajkhoda T., Khanabadi M., Eftekhar M. (2022). PERMA model vs. integrative-behavioral couple therapy for fertility problems: a randomized clinical trial protocol. *International Journal of Reproductive BioMedicine (IJRM)*.

[40] Zdenkowski N., Butow P., Tesson S., Boyle F. (2016). A systematic review of decision aids for patients making a decision about treatment for early breast cancer. *The Breast*.

